The article "A Lightweight Convolutional Neural Network Model for Liver Segmentation in Medical Diagnosis" was published in 2022. Journal: Comput Intell Neurosci.

# A Lightweight Convolutional Neural Network Model for Liver Segmentation in Medical Diagnosis

**DOI:** 10.1155/2022/7954333

**Published:** 2022-03-30

**Authors:** Mubashir Ahmad, Syed Furqan Qadri, Salman Qadri, Iftikhar Ahmed Saeed, Syeda Shamaila Zareen, Zafar Iqbal, Amerah Alabrah, Hayat Mansoor Alaghbari, Sk. Md. Mizanur Rahman

**Affiliations:** ^1^Department of Computer Science and IT, The University of Lahore, Sargodha Campus, Sargodha 40100, Pakistan; ^2^College of Computer Science and Software Engineering, Computer Vision Institute, Shenzhen University, Shenzhen 518060, Guangdong, China; ^3^Computer Science Department, MNS-University of Agriculture, Multan 60650, Pakistan; ^4^Faculty of Information Technology, Beijing University of Technology, Beijing 100124, China; ^5^Department of Computer Science, Ibadat International University, Islamabad 44000, Pakistan; ^6^Department of Information Systems, College of Computer and Information Sciences, King Saud University, Riyadh 11543, Saudi Arabia; ^7^Botany Department, Faculty of Science, Taiz University, Taiz 6803, Yemen; ^8^Information and Communication Engineering Technology, School of Engineering Technology and Applied Science, Centennial College, Toronto, Canada

## Abstract

Liver segmentation and recognition from computed tomography (CT) images is a warm topic in image processing which is helpful for doctors and practitioners. Currently, many deep learning methods are used for liver segmentation that takes a long time to train the model which makes this task challenging and limited to larger hardware resources. In this research, we proposed a very lightweight convolutional neural network (CNN) to extract the liver region from CT scan images. The suggested CNN algorithm consists of 3 convolutional and 2 fully connected layers, where softmax is used to discriminate the liver from background. Random Gaussian distribution is used for weight initialization which achieved a distance-preserving-embedding of the information. The proposed network is known as Ga-CNN (Gaussian-weight initialization of CNN). General experiments are performed on three benchmark datasets including MICCAI SLiver'07, 3Dircadb01, and LiTS17. Experimental results show that the proposed method performed well on each benchmark dataset.

## 1. Introduction

Liver disease is among the most serious medical conditions that can threaten human life and health. Liver tumors are the second primary reason of death in men and the sixth foremost cause of death in females. In 2008, 750,000 people have been identified with liver malignancy and 960,000 people died as a result of the disease [1]. CT scan is a prominent technique for surgical planning and to diagnose organs in the abdomen [2]. Therefore, CT scan is also regularly used to diagnose liver cancer. Liver segmentation is a critical step in computer-aided therapeutic interpolation using CT images, such as volume estimation, radiation, and surgery of liver transplantation. Manual allocation of each slice is a quiet regular clinical rehearsal for the liver description. As a result, manual segmentation is inefficient, independent, and time-consuming. In this manner, creating a fully automated system capable of diagnosing, monitoring, and expediting therapeutic planning is critical. Numerous techniques for segmenting the liver in CT scans have been described, and a summary of these techniques is provided in [3]. Generally, these methods are classified into three classes, which are interactive [4], semiautomatic [5–7], and automatic [8,9]. Interactive and semiautomatic methods depend on a little or a massive user interaction while automatic methods do not depend on any type of user interaction. Semiautomatic approaches have a potential to reduce the effectiveness of a physician.

To date, there are two types of automatic methods frequently used for liver segmentation. Some approaches based on learning and some approaches are based on antilearning including graph cuts [6,10,11], level set [12,13], and region growing [14]. For some challenging datasets, Wang et al. [15] presented a method that defined a shape-prior-level set method to describe the borders of the liver have a level of changeability that is comparable to those which manually achieved. The popular graph cut approaches for the segmentation of the liver are the extension of standard graph cut method proposed by Boyokov et al. [16,17]. Linguraru et al. [18] presented a method for liver segmentation where the generic-affine-invariant shape parametrization method is integrated with the geodesic-active-contour method and segmented a tumor with the graph cut method. The deformable graph cut method is proposed by Li et al. [19] to detect the surface of the liver using the graph cut with a shape constraint. Rusku et al. [14] proposed a neighborhood-connected region growing method that integrated the local neighborhood of the voxels to segment the 3D liver from CT images. In liver segmentation, level set methods are very successful because it can capture complex shapes and also control shape regularity. Using a sparse representation for local and global information of an image, a level set method is proposed by Sheikhli et al. [20]. Atlas-based methods and active shape models (ASMs) are the traditional learning-based methods. Basically, ASM methods first build a shape of the liver and then tie it to the target image. To challenge the task of liver segmentation, Heimann et al. [21] suggested a technique which is the mixture of SSM and a deformable mesh. A probabilistic active contour method is proposed by Wimmer et al. [22], which combined the shape, boundary and region information into an individual level set equation. A multitiered statistical shape model for liver segmentation is proposed by Erdt et al. [23]. For the precise segmentation of hepatic veins, liver, portal veins, and its tumors simultaneously, Wang et al. [24] presented a method using the sparse-shape-composition (SSC) to build a dynamic contour preceding for the liver. The abovementioned active shape model (ASM) performs well on the liver segmentation but it needs a larger dataset and it is also very complicated to build these time-consuming methods. Then registration algorithms are also needed for the correspondence between the liver atlases and their targets. So, these methods are not independent, they need prior knowledge to tackle the segmentation problems. The registration process is also time-consuming and very complicated in terms of liver abdominal CT images. In atlas-based methods, label fusion and selection of atlases are not easy tasks; therefore, these methods have a very limited clinical usage. When the above machine learning methods in the literature are used on challenging cases that have some limitations, especially in liver segmentation which have an irregular shape, the same intensity level in nearby organs (spleen, heart, and right kidney) and tumor in the liver make it more challenging.  Figure 1 shows some of challenges in the CT abdominal images having liver and surrounding organs.

Recently, deep learning approaches have earned considerable interest for their ability to learn a hierarchy of features from high to low [36–39]. A review of different deep learning method for COVID-19 is presented [40–42]. These are very powerful methods as compared to machine learning [43], which can acquire more classified features for image segmentation [44] and classification tasks [45–49]. Qadri et al. [25,26], employing a deep belief network, suggested an approach for segmenting the spine from CT images. Ahmad et al. [27] suggested a system for segmenting the liver using stacked autoencoders that learned unsupervised features. A work based on stacked sparse autoencoder (SSAE) for pedestrian gender recognition achieved outstanding results [28]. Hirra et al. [29] used a deep belief network for breast cancer classification using histopathological images. The skin is segmented using a stacked autoencoder to capture the high-level features [50]. CNN is a form of traditional deep learning technique, which may detect nonlinear mappings between its inputs and outputs [51,52] and visual object recognition [53]. Zhang et al. proposed a two-dimensional convolutional neural network for multimodal infant brain image segmentation [31]. In [54], using a combination of deep learning and graph cut techniques, created a fully automatic system for liver segmentation. It starts with a liver segmentation simultaneously using a probability map learned from a 3D CNN. The graph cut method is used to refine the initial segmentation, and this technique is completely automated and capable of simultaneously learning low-to-high-level features. While [32] presented a deep learning technique called a 3D CNN for automated liver segmentation, which trained and got the subject-specific probability map of the liver that acts as a shape prior and gives the initial surface of the liver. This model is built on the preceding segmentation using local and global information. The global information is used in the healthy part of the liver to learn the area appearance and intensity dissemination, and the local nonparametric information is used to get the abnormal liver information. To resolve the problem of liver segmentation [33], a new 3D convolutional neural network is presented. The suggested model 3D-DSN is better than the simple CNN model in terms of discrimination capability, optimization, efficiency, and effectiveness. 3D-DSN model is a fully convolutional model that is effective in learning. The deep supervision approach to the hidden layer in this work has been used which improve the convergence rate of optimization and increase the precision. To refine the segmentation in postprocessing, a conditional random field is used. Liver and its tumor segmentation are carried out using Octave CNN, which got better results [35,55]. Deep learning methods are being used to detect the tumor from CT images and get reasonable results [56,57]. FCNN was trained on a 3D CT volume of the liver [34], and then a cascade fully convolutional neural network (CFCN) was applied to CT data slices to extract the liver and its lesion. Afterward, 3D-CRF is applied for postprocessing to enhance the segmentation results. Larger parameters, sufficient memory requirements, and extra computational powers are needed in fully 3D convolutional neural network models [58]. To avoid the fully three-dimensional CNN network, two-dimensional patches are utilized and processed these patches for segmentation. The major reason behind it is to discourage the fully 3D CNN because this method is very much expensive in terms of parametric complexity which takes longer time to train the network. So, over segmentation problem might occur due to the biases in rare classes [59].  Table 1 summarizes the recently published deep learning methods. There are some recent deep learning methods which have been used for the detection of different diseases that performed well [60–67].

We extracted the 2D patches from our datasets and processed them with a 2D convolutional neural network to avoid the complexity of fully 3D CNN. Preprocessing is performed to get the enhanced CT image. The input of 2D patches is given to CNN then acquire the probability map:

1. We developed a lightweight convolutional neural network to separate the liver from CT scan images.
2. The proposed CNN model consists of three convolutional and two fully connected layers hence efficiently segmenting the liver.
3. The weights are initialized using a random Gaussian distribution, which does a distance preserving of the information. We added the LRN layer after each convolutional layer to enhance the data adaptability.
4. Three benchmark datasets SLiver'07, 3Dircadb01, and LiTS17 are used to analyze the model performance which improves the stability of our model.

The whole article is organized as follows: Sections 2–4 are the proposed method, experimental setup, and results and discussion, respectively. The conclusion is given in Section 5.

## 2. Proposed Method

This section provides details of the method we followed in this study. The whole pipeline of our system is illustrated in Figure 2.

### 2.1. Data Preparation

A simple preprocessing is applied in the proposed work on each axial CT slice. We enhanced the contrast and normalized the dataset using zero mean and unit variance to obtain the data range between 0 and 1. On both the training and testing datasets, we applied similar steps. For the training dataset, we applied the additional step to augment the input data. We crop the train data where liver slices are not affected and rotate the images on 90, 180, and 270°. The detail of data augmentation is given in the literature [68,69]. We sliced each axial 2D image into 32 × 32 patches for both training and testing data and picked 1.3 million patches from the background and foreground randomly for training data. The image patches of two classes are equally taken with a ratio of 1 : 1 for stable training and validation.

### 2.2. Convolutional Neural Network

We briefly discuss the convolutional neural network (CNN) in this section. More detail on CNN can be found in [51,70]. The CNN is a discrepancy of a multilayer perceptron. The core part of CNN is based on convolutional and subsampling layers. For the hierarchy of feature learning in the convolutional neural network, numerous convolutional layers are heaped together. Every convolutional layer is capable of obtaining the feature map from the layer before it. These layers are connected with some filters. We indicate that Con^(*n* − 1)^ and Con^(*n*)^ are the input and output of the *n* convolutional layers, respectively, and Con_*i*_^(*n*)^ denotes *i*th feature map of the *n*^th^ layer in a particular CNN. The following equation can be used to calculate the output of the *n*th layer.

(1) $$\begin{array}{c} C_{j}^{\left(m\right)}=\;F_{W,\;b}\left(\underset{i}{\sum }C_{i}^{n-1}*\;W_{i,j}^{\left(n\right)}b_{j}^{n}\right). \end{array}$$

Here, *W*_*i*,*j*_^(*n*)^ is the kernel relating of *i*th and *j*th output map and *∗* is the denotation of the convolution and *b*_*j*_^*n*^ denotes the bias of the *j*th output record of the *n*th layer in a particular convolutional layer. *F*_*W*, *b*_(.) denotes a nonlinear activation function. For nonlinear activation, the function has many options, which are rectified linear unit (ReLU), sigmoid, and hyperbolic tangent. A subsampling layer after the convolutional layer is used to reduce the computational complexity. So, in this manner, we adapt the max-pooling layer which is commonly used. Fully connected layers are often used after the convolutional layers and at the end, a softmax classifier is used to classify the results. In binary classification problems, the regression model is being used to normalize the results of kernel convolution. Convolutional layers are sharing the weights which is the key advantage of CNN. Each pixel in the layer uses the same filter. The main advantage is to improve the performance as well as reduce the memory size.

If the training set is made up of *m* labeled samples,

 
{(*x*^1^,  *y*^1^),  (*x*^2^,  *y*^2^),…, (*x*^*m*^,  *y*^*m*^) }, *y*^*i*^  can be 0 or 1, where *I* = (1, 2, 3,…, *m*).

*θ* indicates all the important parameters including bias, kernel, and softmax parameters of the CNN. Concerning  *θ*, we reduce the following cost function for logistic regression.

(2) $$\begin{array}{c} E\left(0\right)=-\frac{1}{m}\left[\overset{m}{\underset{i=1}{\sum }}y^{i}\log\;F_{\theta }\left(x^{i}\right)+\left(1-y^{i}\right)\log\left(1-F_{\theta }\left(x^{i}\right)\right)\right]. \end{array}$$

For regularization of classification, weight decay can be used to castigate the larger values of the softmax layer. Gradient-based optimization can be utilized to reduce the cost function [52] and backpropagation is used to calculate the partial derivatives [51].

### 2.3. Proposed Ga-CNN Architecture

For any low-dimensional data, random estimation is a general sampling approach [71–73]; a deep neural network with random weights is a general system that can separate the data. The angles among its points, it is observed that there are larger angles among different classes [74–77]. The intraclass angles are more important than interclass ones in a deep network.

The recent study shows that the vital property of Gaussian distribution is to preserve the ratio among the angles in the data during the DNN training. Therefore, it does not give a priority in any direction but it treats the same to each direction; the above discussion is leading to the behavior of distances and angles throughout the DNN net. In common, there are small angles between the points in the same class but have a larger distance in different classes. Random Gaussian weights would be a good choice for the DNN network parameters if it holds all the points. We adopted the random Gaussian weights for the initialization of the training network, where the hypothetical details and proofs are given in the literature [78]. To address the problem of liver segmentation in CT images, a patch-based methodology is being developed. The first 2D image is separated into *M* number of patches. The input image of axial slice with size of 512 × 512 is divided into 1 × 32 × 32 patch size, where 1 is the channel of the image patch.  Figure 3 shows the foreground and background patches.

The proposed DNN method has the input of 1 × *N* × *N* 2D patch of CT scan images. The most important and necessary layer for building the CNN model is a convolutional layer. Numerous convolutional layers are placed on top of one another to create a feature hierarchy. Each layer receives its input from the layer that was previously connected. The convolutional layer executes the stack of input CT image patches and outputs the number of feature maps. Each region of interest corresponds to a topological arrangement inside the responsive map of a specific nonlinear spatial feature abstraction. These learning parameters could very certainly be applied to any spatial neighborhood layout using the sliding window architecture. The convolutional layer activation process is dependent on the single plan of an input CT image. The feature map from previous layers is often included in the information plan for subsequent layers. In the proposed model, we are using three convolutional and two fully connected layers. Convolutional layers are the main components of CNN, reducing the number of dimensions while increasing the depth. The filter size of 7 × 7 in the first, 5 × 5 in the second, and 3 × 3 in the third convolutional layer are used.  Figure 4 shows the proposed Ga-CNN network architecture. The other information regarding each layer in our model is given in Table 2.

Each convolutional layer is tailed by a ReLU, LRN, and max-pooling layer. Our network contains three max-pooling layers, where 3 × 3 sub-window size is being used with stride of 2 in the first and second max-pooling layers and a sub-window size of 2 × 2 with a stride of 2 is used in every path of third max-pooling layer [79]. ReLU is a piecewise linear transformation max (*x*, 0) that improves convergence by selecting important invariant features that enhance the execution's generality [51]. ReLU has a required property that does not need any input normalization to stop them from soaking. If a positive input is produced by a training example that is given to ReLU, that neuron will be learned. Therefore, LRN still adds the generalization. The following formula is used to calculate the LRN.

(3) $$\begin{array}{c} b_{x,y}^{i}=\frac{x}{K+\alpha \sum_{j=\text{max}\left(0,\;i-N/2\right)}^{\text{min}\left(N-1,\;I+N/2\right)}{\left(a_{x,y}^{j}\right)}^{2}{\;}^{\beta }}, \end{array}$$

where *b*_*x*,*y*_^*i*^ is the response normalization activity, where the sum runs across N neighboring kernel maps and the layer comprises N number of kernels at the same spatial position. We used the same LRN hyperparameters as in [51]. The convolutional layer produces the output of the feature mapping procedure as an input from the preceding convolutional layer. From the perspective of the neural network, feature maps are associated with the hidden layers of neurons. Each coordinate subset of features is associated with a single neuron, and the size of the receptive field is proportional to the kernel size. Finally, at the network's end, two fully connected layers are added. The fully connected layer executes the scalar product, where the input is a vector and it returns a scalar. The first fully connected layer with a neuron size of 4096 and the dropout factor of 0.3 is used. Dropout is employed during the training phase to keep the network from overfitting. The second fully connected layer which is final layer of our system, and then softmax classifier is used to perform classification for our model (Background and Liver). We reconstructed the image on the bases of classification results to perform a segmentation. Meanwhile, after segmenting each 2D liver image, we used a 5 × 5 median filter to smother the resultant liver. Total trainable parameters of our model (Ga-CNN) are about 10 million; if we compare these parameters with Alexnet, which has 62 million, and VGG16, they are about 138 million. In terms of complexity, our model is less complex and stable. The information of trainable parameters is given in Table 2.

## 3. Experimental Setup

In total, 60 contrast-enhanced CT images with ground truths were used to train the network. We used three challenging datasets in our work, which are the SLiver'07 training set, 3Dircadb01, and LiTS17 training dataset. We have selected 10 CT images from the SLiver'07 training set, 10 CT images from 3Dircadb01, and 40 CT images from the LiTS dataset for training and validation. All three benchmark datasets are freely available online. In total, 30 contrast-enhanced CT images were selected for testing purposes, where the axial slice resolution was 512 × 512 pixels. We randomly selected 10 CT images from SLiver'07, 10 CT images from 3Dircadb01, and 10 CT images from the LiTS17 dataset. For experiments, we adopted the MATLAB 2021a for implementation of our model. We selected the parameters which are Stochastic Gradient Descent with Momentum (SGDM) and initial learning rate of 0.01 for this experiment. A computer with windows operating system, Intel Core i-7, 8565U processor, 32 GB of RAM with 2 GB GPU (NVIDEA GeForce 250) was used.

In our method, we initialized the weights manually from a Gaussian distribution with a standard deviation of 0.0001. We applied Gaussian weights to CNN network which perform steady inserting of the input data that draw a linking among the features produced by our model [78]. We trained our model with 70 epochs where we set the initial learning rate of 0.01. After 20 epochs, the learning rate dropped by a factor of 0.1. Momentum was constant in the whole experiment, which was 0.9. Weight decay and mini-batch size were 0.0001 and 64, respectively. Stochastic gradient descent with momentum (SGDM) is used as an optimization algorithm. The SGD algorithm has trouble, where the surface curve is much tighter in one dimension than another [80]. Momentum is the method that can help the SGD to accelerate in a relevant direction [81]. The training hyperparameters are given in Tables 3 and 4. The proposed model performance is analyzed by key modules that affect and extract the patches.  Figure 5 shows the visualization of three convolutional layers in our training model.

After the training, the trained CNN algorithm is learned iteratively from the initial liver probability map. One of the test volumes in Figure 6 shows the iterative results of the liver probability map. In the 8^th^ iteration, the liver and spleen had the same intensity and texture level but in the 15^th^ iteration, the liver becomes brighter which means liver pixels are stronger and easily differentiable. In a 25^th^ iteration, the spleen becomes smaller as in previous iterations. In the 35^th^ iteration, the spleen disappeared and the liver becomes brighter. In the 60^th^ to 70^th^ iterations, the validation results converge and the shape of the liver becomes accurate.

## 4. Results and Discussion

In this section, we provide the detailed segmentation results based on three benchmark datasets which are SLiver'07, 3Dircadb01, and LiTS17. The input image is converted into multiple 2D patches and given as an input to Ga-CNN model for detection and then segmentation is performed on the input image.

All the three benchmark datasets (having normal and abnormal CT scan images) are evaluated on eight performance metrics such as SE, SP, ACC, Precision, FPR, FNR, JSI, and DSC. In equations 4 to 11, true positive (TP) denotes all the pixels related to the liver, true negative (TN) shows all the pixels related to the background. False negative (FN) denotes the liver pixels that do not classify accurately, and false positive (FP) denotes the pixels which belong to the background but are not identified as a background. The dice similarity coefficient (DSC) is being used for the calculation of automatic and manual segmentation, and JSI is used to measure the similarity between the two images.

(4) $$\begin{array}{c} \text{SE}=\frac{\text{TP}}{\text{TP}+\text{FN}}, \end{array}$$

(5) $$\begin{array}{c} \text{SP}=\;\frac{\text{TN}}{\text{TN}+\text{FP}}, \end{array}$$

(6) $$\begin{array}{c} \text{ACC}=\frac{\text{TP}+\text{TN}}{\text{TP}+\text{TN}+\text{FP}+\text{FN}}, \end{array}$$

(7) $$\begin{array}{c} \text{Precision}=\frac{\text{TP}}{\text{TP}+\text{FP}}, \end{array}$$

(8) $$\begin{array}{c} \text{FPR}=1-\text{Specificity,} \end{array}$$

(9) $$\begin{array}{c} \text{PNR}=1-\text{Sensitivity,} \end{array}$$

(10) $$\begin{array}{c} \text{JSI}=\frac{\text{DSC}}{2-\text{DSC}}, \end{array}$$

(11) $$\begin{array}{c} \text{DSC}=\frac{2\text{TP}}{\text{FP}+2\text{TP}+\text{FN}}. \end{array}$$

The analysis of key components is analyzed which affect and extract patches on the proposed model. In this section, previous deep learning and machine learning methods are being compared. Finally, the outcomes of three benchmark datasets are conveyed by experimentation.

We presented the results of 10 CT images that were randomly selected out of 20 CT images for testing purpose in Sliver'07 dataset. The overall DSC of 95.0%, Jaccard similarity index of 90.47%, the accuracy of the proposed model of 95.1%, precision of 97.2%, sensitivity of 95%, specificity of 95.2%, FNR of 0.048, and FPR of 0.05 are noted on the SLiver'07 dataset. We observed from the above results that our method performed well in classification as well as in segmentation.  Figure 7 depicts the segmentation results on 2D axial slices of the SLiver'07 dataset on the proposed model. The axial slices are randomly chosen from different CT images of the SLiver'07 dataset. Segmentation results show that the proposed model efficiently recognized the boundaries of the liver, where (a) is the original CT image, (b) is the original label, (c) is the segmentation results of Ga-CNN model, and (d) is the overlapping results of the original label (green) and segmented results of Ga-CNN (red).

The qualitative results of 3Dircadb01 datasets are presented in Table 6. 3Dircadb01 dataset composed of 20 CT images; we presented the mean results of 10 CT images, which were selected from 3Dircadb01 dataset randomly for testing. The DSC of 92.9%, JSI of 85.1%, the accuracy of the proposed model of 93.1%, precision of 95.5%, sensitivity of 93.0%, specificity of 93.2%, FNR of 0.08, and FPR of 0.07 are noted on the 3Dircadb01 dataset.  Figure 8 shows the segmentation results on 2D axial slices of the former dataset on the proposed model. The axial slices are randomly chosen from different CT images of the 3Dircadb01 dataset, where (a) is the original CT image, (b) is the original label, (c) is the segmentation results of Ga-CNN model, and (d) is the overlapping results of original label (green) and segmented results of Ga-CNN (red).

We presented the mean results of 10 CT images which were selected from LiTS dataset randomly in Table 7. The DSC of 97.31%, JSI of 94.76%, the accuracy of the proposed model of 97.25%, precision of 97.06%, sensitivity of 97.56%, specificity of 96.93%, FNR of 0.02, and FPR of 0.02 are noted on LiTS dataset. The axial slices are randomly chosen from different CT images of LiTS dataset.  Figure 9 shows the results of LiTS17 dataset, where (a) is the original CT image, (b) is the original label, (c) is the segmentation results of Ga-CNN model, and (d) is the overlapping results of original label (green) and segmented results of Ga-CNN (red).

The intermediate results of all the three datasets are given in Table 8. The mean DSC of 95.07%, JSI of 90.65%, ACC of 95.15%, precision of 96.58%, SE of 95.18%, SP of 95.11%, FNR of 0.05, and FPR of 0.05 are noted. The overall performance of the proposed model is better and can be comparable to another state-of-the-art methods in the literature.  Table 9 depicts the comparison of the proposed method results with other recently published well-known liver segmentation methods.

The comparison with other recently published liver segmentation methods is given in this section. In [82], liver segmentation is performed on CT images using two challenging datasets which are 3Dircadb01 and SLiver'07. DSC of SLiver'07 and 3Dircadb01 datasets are 94.03% and 91.19%, respectively. This method is somewhat complex and needs to remove the rib from the CT image and then apply the random walker algorithm to extract the liver but the proposed method do not need to remove any other organ first. Ga-CNN detects the liver boundaries very efficiently without any other postprocessing support. If we compare our method with that in [35], the DSC of our method is 95.07% which is better. We conducted the experiments on three benchmark datasets with 30 contrast-enhanced CT images, that can also validate our algorithm. Another recently published deep learning method using a stacked autoencoder (DSAE) [27] got 90.1% DSC that is less than the proposed method. The training and validation of Deep stacked auto encoder (DSAE) are performed on 2 publicly available datasets (3Dircadb and Sliver'07); the limitations of this method against our methods are obvious that DSAE cannot detect the abnormal liver in the image very well but our method can efficiently segment the abnormal liver very efficiently. In [46], the DSC of liver segmentation was noted 92% using LiTS17 dataset that is less than the DSC in our proposed work. In [35], the two datasets, SLiver'07 and 3Dircadb01, that were used to segment the liver show the DSC of 94.80% and 91.83%, respectively, which are obviously much fewer than Ga-CNN method. Proposed algorithm has a capability to find the edges and curves very accurately, and the computational time for each slice is only 6 seconds, which shows that Ga-CNN is very lightweight. The application of our method is best for the donors of the liver, because the normal liver can be efficiently segmented with correct boundaries. From the segmentation results shown in Figures 7–9, it is clearly observed that the proposed method correctly segments the areas of the liver from the CT images, where the heart, stomach and spleen also having the same intensity level. Normally, the spleen and stomach are mis-segmented by many algorithms because of their same intensity nature, but our DNN correctly identifies the liver pixels and discriminates the other organs due to the efficient feature learning. Liver shape variability is also a big problem in CT images but our algorithm can solve it effectively.

In the above discussion, we compared our method with deep learning and some other liver segmentation methods. We observed the above given experimental results that the proposed technique is better as compared to the other recent methods in the literature. This proves the applicability of the proposed method. The validation results of three well-known benchmark datasets also make our algorithm very proficient. Overall, we found in our research that initialization of DNN with random Gaussian weights perform better and have a steady insertion of a data. The most important is to draw the connection among the dimensions that are generated by the DNN and still retain the complication of the data and matric information of the original manifold. The results of the proposed method show that deep neural networks are general classifier for that data which is based on the angles of major alliance among the classes in the data. Our random Gaussian initialization is mainly focused on the previous study that proved that this strategy is also better to train the DNN models with low training samples. For liver segmentation, this also helps us improve the results of the abnormal liver, where the angles and shapes of the liver could be detected in a better way. The 3Dircadb01 and LiTS are both complex datasets, having different types of tumors in it. But the mean DSC and precision of these two datasets prove that our proposed model performed well and can be approachable against other well-known methods.

## 5. Conclusion and Future Work

This study proved the development of an accurate and robust technique of a liver segmentation. The developed algorithm accomplished the segmentation with a very light convolutional neural network (Ga-CNN) with randomly initialized Gaussian weights, which performed a steady insertion of the data that draw the linking between the magnitudes of the features produced by our network that still preserve the metric evidence of the complexity of the data and the original manifold. Adding ReLU activation function after each convolutional layer makes the learning very fast and found early convergence. Also, we introduced local response normalization (LRN) after ReLU which improved the precision and reduced the false positive rate. The validation of three benchmark datasets including SLiver'07, 3Dircadb01, and LiTS17 prove that the proposed model performed better on CT images to segment the liver. The recorded mean dice, Jaccard index, accuracy, and precision were 95.07%, 90.65%, 95.15%, and 96.58%, respectively, on 30 CT test images.

We tested our model on three datasets, which gives better accuracy and DSC. On the bases of these results, we are sure that our lightweight CNN could give better results for the segmentation of liver with other datasets. In future, we will add more dataset for more accuracy. Moreover, our method could be applied on other organs for segmentation, like the kidney, lungs, and heart. Our lightweight CNN model is limited for the segmentation of a liver. On complex datasets like 3Dircadb01, the accuracy of Ga-CNN is less than other used datasets. For this purpose, we will improve our preprocessing techniques to cope this situation. We will also focus on liver tumor segmentation using Ga-CNN with more improvements.

## Figures and Tables

**Figure 1:** Sketch of challenges in automatic liver segmentation. The shape of the liver changes in different cases. Nearby organs have a similar intensity level.

**Figure 2:** Flow diagram of our methodology.

**Figure 3:** The foreground and background patches. Each patch size is 32 × 32 pixels, and *M* is the total number of extracted patches.

**Figure 4:** Proposed Ga-CNN architecture.

**Figure 5:** Visualization results of filters of each convolutional layer. The 1^st^ convolutional layer with 32 filters, the 2^nd^ convolutional layer with 192 filters, and the 3^rd^ convolutional layer with 256 filters.

**Figure 6:** Iterative results of liver probability map produced by Ga-CNN model on CT scan image of SLiver'07 dataset. From top left to bottom right, 8^th^, 15^th^, 25^th^, 55^th^, 60^th^, and 70^th^ iterative liver probability maps are shown. The brighter region shows the more probability map of the liver.

**Figure 7:** The results of segmentation of SLiver'07 dataset.

**Figure 8:** The results of segmentation of 3Dircadb01 dataset.

**Figure 9:** The results of segmentation of LiTS dataset.

**Table 1:** The recently published deep learning methods to perform different classification and segmentation tasks.

S. no.	Author	Technique name	Purpose	Date published
1	Qadri et al. [25]	Deep belief network with two hidden layers	Deep belief network is used for the spine segmentation from CT images.	2018
2	Qadri et al. [26]	Pa-DBN with two hidden layers	Employing a deep belief network, suggested an approach for segmenting the spine from CT images.	2019
3	Ahmad et al. [27]	DSAE with two hidden layers	Segmenting the liver from CT images using stacked autoencoders that learned unsupervised features.	2017
4	Raza et al. [28]	Stacked sparse autoencoder (SSAE)	HOG-based features generated and then sparse stacked autoencoder is used for pedestrian gender recognition.	2018
5	Hirra et al. [29]	Pa-DBN-BC	Deep belief network for breast cancer classification using histopathological images.	2021
6	Lei et al. [30]	Stacked autoencoder	The skin is segmented using a stacked autoencoder to capture the high-level features.	2016
7	Zhang et al. [31]	CNN with three convolutional and a fully connected layer is used; after the convolutional layer, local response normalization layer is used	Propose a two-dimensional convolutional neural network for multimodal infant brain image segmentation.	2015
8	Hu et al. [32]	3D CNN	Presented a deep learning technique called a 3D CNN for automated liver segmentation which trained and got the subject-specific probability map of the liver that acts as a shape prior and gives the initial surface of the liver.	2016
9	Dou et al. [33]	3D-DSN	The suggested model 3D-DSN is better than the simple CNN model in terms of discrimination capability, optimization, efficiency, and effectiveness.	2016
10	Christ. et al. [34]	FCNN	FCNN is trained on a 3D CT volume of the liver and then a cascade fully convolutional neural network (CFCN) was applied to CT data slices to extract the liver and its lesion. Afterward, 3D-CRF is applied for postprocessing to enhance the segmentation results.	2017
11	Ahmad, et al. [35]	DBN-DNN	Liver segmentation is performed from CT images using deep belief network. This method gives good accuracy and DSC.	2019

**Table 2:** The CNN model's detailed architecture is employed in this work.

Type of layer	Kernel	Stride	Padding	Output	Depth	Trainable parameters
Input	—	—	—	32 × 32	1	
Convolution	7	2	0	13 × 13	32	1600
Max-Pooling	3	2	0	13 × 13	32	0
Convolution	5	1	2	13 × 13	192	153792
Max-Pooling	3	2	0	6 × 6	192	0
Convolution	3	1	1	6 × 6	256	442624
Max-Pooling	2	2	0	3 × 3	256	0
Fully connected	1	—	—	1 × 1	4096	9,441,280
Fully connected	1	—	—	1 × 1	2	8,194
Softmax	—	—	—	1 × 1	2	
Total						10,047,490

**Table 3:** Hyperparameters of Ga-CNN.

Parameter	Value
Momentum	0.9
L2 Regularization	0.0001
Max epochs	70
Mini-batch size	64

**Table 4:** Learning rate schedule.

Learning rate	Value
Initial	0.01
Schedule	Piecewise
Drop factor	0.1
Drop period	20

**Table 5:** The segmentation results of SLiver'07 training dataset using the proposed model.

Dataset	DSC%	JSI%	ACC%	Precision%	SE%	SP%	FNR	FPR
SLiver'07	95.0	90.47	95.1	97.2	95	95.2	0.048	0.05

**Table 6:** The segmentation results of the 3Dircadb01 dataset using the proposed model.

Dataset	DSC%	JSI%	ACC%	Precision%	SE%	SP%	FNR	FPR
3Dircadb01	92.9	86.74	93.1	95.5	93.0	93.2	0.08	0.07

**Table 7:** The segmentation results of LiTS17 training dataset using the proposed model.

Dataset	DSC%	JSI%	ACC%	Precision%	SE%	SP%	FNR	FPR
LiTS17	97.31	94.76	97.25	97.06	97.56	96.93	0.02	0.03

**Table 8:** The intermediate results of the proposed model on three benchmark datasets.

Dataset	DSC%	JSI%	ACC%	Precision%	SE%	SP%	FNR	FPR
SLiver'07	95.00	90.47	95.10	97.20	95.00	95.20	0.048	0.05
3Dircadb01	92.9	86.74	93.10	95.50	93.00	93.20	0.08	0.07
LiTS17	97.31	94.76	97.25	97.06	97.56	96.93	0.02	0.03
Mean	95.07	90.65	95.15	96.58	95.18	95.11	0.05	0.05

**Table 9:** The comparison with other methods.

Method	Test dataset (s)	DSC%
Random Walker [82]	3Dircadb01	91.19
Random Walker [82]	SLiver'07	94.03
DSAE [27]	3Dircadb01, SLiver'07	90.10
VNET and WGAN [46]	LiTS17	92.00
DBN-DNN [35]	SLiver'07	94.80
DBN-DNN [35]	3Dircadb01	91.83
Proposed	3Dircadb01, SLiver'07, and LiTS17	95.07

## Data Availability

The data supporting the findings of this study are included within the article.
